This article has been retracted.

# Levels of Serum sST2, MMP-3, and Gal-3 in Patients with Essential Hypertension and Their Correlation with Left Ventricular Hypertrophy

**DOI:** 10.1155/2021/7262776

**Published:** 2021-10-12

**Authors:** Xueling Wang, Wei Han, Lin Han, Jiyuan Yang, Kehui Li, Yun Fan

**Affiliations:** ^1^Department of Cardiovascular Medicine, Beijing Hospital of Integrated Traditional Chinese and Western Medicine, Beijing 100039, China; ^2^Department of Cardiology, Beijing Luhe Hospital Affiliated to Capital Medical University, Beijing 101149, China; ^3^Department of Cardiology, Beijing Traditional Chinese Medicine Hospital Affiliated to Capital Medical University, Beijing 100010, China

## Abstract

Essential hypertension (EH) is a clinically frequent cardiovascular disease, with insidious onset, causing increased pressure load and neuroregulation disorders in patients. Long-term EH can cause left ventricular hypertrophy (LVH), which can lead to arrhythmia and even death. The soluble suppression of tumorigenicity 2 (sST2), matrix metalloproteinase-3 (MMP-3), and galectin-3 (Gal-3) in serum plays an important role in the occurrence, development, and prognosis of cardiovascular diseases. In our study, we divided EH patients into 3 levels and groups with or without LVH, according to their condition. The levels of sST2, MMP-3, and Gal-3 in the serum were measured in different groups of patients. Our results showed that the levels of sST2, MMP-3, and Gal-3 in the serum increased progressively with the level in different EH groups. The levels of sST2, MMP-3, and Gal-3 in the serum of the LVH group were higher than those of the NLVH group, and it is positively correlated with LVH-related indexes. The risk of developing and progressing to LVH in patients with EH can be determined by the method of measuring three indicators.

## 1. Introduction

The essential hypertension (EH) is a clinically frequent cardiovascular disease with insidious onset and protracted course. As the disease progresses, essential hypertension can cause damage to multiple organs, cause serious adverse events such as heart failure and stroke, and affect the quality of life of patients [1, 2]. According to the survey, the number of patients suffering from hypertension in 2019 was approximately 245 million, and the prevalence is increasing year by year in my country [3]. The EH patients are prone to left ventricular hypertrophy (LVH) due to increased pressure load and neuromodulation disorders, which seriously harms the prognosis of patients [4]. With the aging of society, the probability of EH patients with LVH gradually increases, which can be as high as 19.2%–34.3% [5]. Therefore, it is necessary to use reasonable indicators to judge the risk of developing LVH in EH patients clinically.

The soluble suppression of tumorigenicity 2 (sST2) is a receptor of the interleukin 1 family, which can regulate the body's immune response and play an important role in events such as myocardial fibrosis and cardiac insufficiency [6]. Zhang et al. [7] conducted a prospective study of 414 maintenance hemodialysis patients and found that, during a median follow-up of 22.3 months, 58 patients died, of which 31 died of cardiovascular disease. sST2 was an independent predictor of death from all causes, with a relative risk value of 1.31 (95% CI 1.000–1.717), and sST2 was also an independent predictor of death from cardiovascular diseases, with a relative risk value of 2.10 (95% CI 1.507–2.927). sST2 has good a prognostic evaluation value in patients with hemodialysis.

The matrix metalloproteinase-3 (MMP-3) is a member of the MMPs' family, which is involved in tissue remodeling and can affect the occurrence and prognosis of a variety of cardiovascular diseases [8]. Hu et al.[9] selected 200 patients with carotid atherosclerosis (CAS) as the study subjects, and another 60 healthy people were selected as the control group, and all subjects were tested for MMP-3 levels. Finally, it was found that compared with healthy people, patients with CAS had higher levels of MMP-3, and the level of MMP-3 in the vulnerable plaque group was significantly higher than those in the stable plaque group and the nonplaque group. MMP-3 was positively correlated with cardiovascular and cerebrovascular events in patients with CAS, which could be used as a marker for the clinical diagnosis and prognosis assessment of patients with CAS.

The galectin-3 (Gal-3) is a member of the galectin family and plays a key role in the diagnosis of myocardial infarction, heart failure, and other diseases [10]. Martínez-Martínez's et al. [11] believed that myocardial fibrosis is the main factor leading to heart failure. The levels of myocardial Gal-3 and plasma Gal-3 in the body of patients with heart failure increased significantly. The higher the level of Gal-3, the higher the risk of cardiovascular death in patients with heart failure; Gal-3 has become a candidate therapeutic target and prognostic evaluation indicator of heart failure.

At present, there is no clinical research report on the correlation between the levels of sST2, MMP-3, Gal-3, and LVH. The aim of this study was to investigate the serum sST2, MMP-3, and Gal-3 levels in EH patients and to analyze their correlation with LVH.

## 2. Materials and Methods

### 2.1. General Materials

267 patients with EH were selected for treatment from March 2019 to March 2020. There were 145 males and 122 females, ranging in age from 23 to 81 years old, with an average age of (54.25 ± 8.63) years old; there were 114 cases of diabetes and 81 cases of hyperlipidemia. Inclusion criteria: the patient met the EH diagnostic criteria [12], all EH patients had been taking antihypertensive drugs regularly, and no family history of EH. Exclusion criteria: secondary hypertension, congenital heart disease, severe liver and kidney dysfunction, malignant tumor, recent history of infection, immune system disease, pregnant and lactating women, and mental illness. In addition, 100 cases of healthy physical examination during the same period were selected as the control group, of which 53 were males and 47 were females and aged 20–79 years old, with an average age of (52.77 ± 8.12) years old; there were 38 cases of diabetes and 25 cases of hyperlipidemia. There was no statistically significant difference in the general information of the two groups (*p* > 0.05), and it was comparable.

According to the grading standard of the guideline, the EH patients were divided into 121 cases in the level 1 EH group, with systolic blood pressure 140–159 (mmHg) and/or diastolic blood pressure 90–99 (mmHg), 87 cases in the level 2 EH group, with systolic blood pressure 160–179 (mmHg) and/or diastolic blood pressure 100–109 (mmHg), and 59 cases in the level 3 EH group, with the systolic blood pressure not less than 180 mmHg and/or the diastolic blood pressure not less than 110 mmHg. According to the presence or absence of LVH, EH patients were divided into 102 cases in the LVH group and 165 cases in the NLVH group. The course of the LVH group was (10.47 ± 5.96) years. The course of the NLVH group was (10.12 ± 6.33) years. There was no statistically significant difference in the general information of each group (*p* > 0.05), and it was comparable. This study was approved by the ethics committee of our hospital, and all the study subjects signed an informed consent form.

### 2.2. Research Methods

4 mL of fasting venous blood was drawn from all study subjects and stored at −80°C after centrifugation. Enzyme-linked immunosorbent assay was used to detect serum sST2, MMP-3, and Gal-3 levels. The relevant test kit was purchased from Beijing Biolab Technology Co., Ltd. The experiment operation was carried out in strict accordance with the instructions. The cardiac ultrasound examination was performed using the U.S. Philips IU22 color Doppler ultrasound diagnostic instrument with a probe frequency of 2–4 MHz, and the average of 3–5 cardiac cycles was taken. The thickness of the ventricular septum (IVST), the thickness of the left ventricular posterior wall (LVPWT), and the end-diastolic diameter of the left ventricle (LVD) was measured, and the left ventricular weight (LVM) was calculated according to De. Vereux correction formula, LVM = 1.04^*∗*^[(IVST + LVPWT + LVD)^3^-LVD^3^]-13.6, LVMI (g/m^2^) = LVM/body surface area, and body surface area = 0.0061^*∗*^height (cm) + 0.0128^*∗*^body weight (kg)-0.1529. The age and body mass index (BMI) of EH patients = weight (kg)/height (m)^2^, systolic blood pressure, diastolic blood pressure, fasting blood glucose, total cholesterol (TC), triacylglycerol (TG), sST2, MMP-3, Gal-3, and other clinical data were recorded, and the risk factors of LVH in EH patients were analyzed.

### 2.3. Statistical Methods

The data of this experiment were statistically analyzed by SPSS22.0. The measurement data were expressed as ($\bar{x}$ ± s), and the comparison adopted *t*-test or analysis of variance. The logistic regression analysis was used for risk factors. The Pearson correlation analysis was used to correlation analysis. The *p* value less than 0.05 indicated that the difference was statistically significant.

## 3. Result

### 3.1. Comparison of Serum sST2, MMP-3, and Gal-3 Levels between EH Group and Control Group

The levels of serum sST2, MMP-3, and Gal-3 in the EH group were higher than those in the control group, and the differences were statistically significant (*p* < 0.05), as shown in Figure 1.

### 3.2. Comparison of Serum sST2, MMP-3, and Gal-3 Levels in Patients with Different Levels of EH

The serum levels of sST2, MMP-3, and Gal-3 in the level 2 and level 3 EH groups were higher than those in the level 1 EH group. The levels of serum sST2, MMP-3, and Gal-3 in the level 3 EH group were higher than those in the level 2 EH group, and the differences were statistically significant (*p* < 0.05), as shown in Figure 2.

### 3.3. Comparison of Serum sST2, MMP-3, and Gal-3 Levels between LVH Group and NLVH Group

The levels of serum sST2, MMP-3, and Gal-3 in the LVH group were higher than those in the NLVH group, and the differences were statistically significant (*p* < 0.05), as shown in Figure 3.

### 3.4. Risk Factors for the Development of LVH in Patients with EH

High systolic blood pressure, high diastolic blood pressure, high levels of sST2, high levels of MMP-3, and high levels of Gal-3 were all independent risk factors for the development of LVH in patients with EH (*p* < 0.05), as shown in Table 1.

### 3.5. Correlation between the Levels of Serum sST2, MMP-3, Gal-3, and LVMI

The levels of sST2, MMP-3, and Gal-3 in serum were positively correlated with LVMI (*r* = 0.638, *p* < 0.01; *r* = 0.446, *p*=0.029; *r* = 0.597, *p* < 0.01), as shown in Table 2.

## 4. Discussion

In recent years, the incidence of EH has gradually increased, causing harm to patients' health and social stability. Long-term EH can cause the heart to become overloaded, resulting in structural changes to the heart and LVH, which can lead to arrhythmias, strokes, and even death [13, 14]. Therefore, finding risk factors for the development of LVH in patients with EH is important to improve the prognosis of patients.

As a commonly used clinical marker, sST2 plays a key role in protecting cardiomyocytes, regulating the body's inflammatory response and immune response, which can also evaluate ventricular remodeling and heart failure [15, 16]. Parikh et al. conducted a survey of 3915 elderly people and found that the higher level of sST2 were associated with a higher the risk of heart failure, myocardial damage, and myocardial fibrosis. sST2 can effectively predict cardiovascular death in the elderly [17]. Due to its ability to degrade collagen and activate other MMPs, MMP-3 can affect the occurrence and development of the EH patients and play an essential role in tissue remodeling, causing diastolic dysfunction in the heart and endangering the health of patients [18]. The Gal-3 participates in cell growth, proliferation, and apoptosis of the body and is a common clinical test index. The level of Gal-3 is low in healthy people, while in patients with myocardial damage, its level rises rapidly, which has a good predictive value in the pathological development of EH [19, 20]. In this study, the serum levels of sST2, MMP-3, and Gal-3 in the EH group were higher than those in the control group, and the level 2 and level 3 EH groups were higher than those in the level 1 EH group, and the level 3 EH group were higher than those in the level 2 EH group. The results showed that the levels of sST2, MMP-3, and Gal-3 in the serum of EH patients increased, and they increased with the aggravation of EH disease.

The results of this study also showed that the serum levels of sST2, MMP-3, and Gal-3 in the LVH group were higher than those in the NLVH group. High systolic blood pressure, high diastolic blood pressure, high level of sST2, high level of MMP-3, and high level of Gal-3 were all independent risk factors for LVH in the serum of EH patients. The levels of sST2, MMP-3, and Gal-3 in the serum were positively correlated with LVMI. This means that the levels of sST2, MMP-3, and Gal-3 in the serum of EH patients were closely related to LVH. The possible reason is that the shear stress of the blood flow to the blood vessel wall in EH patients was increased, endothelial cells were damaged, and the tension of the blood vessel wall was increased, which in turn endangered the patient's heart function [21]. EH patients have high systolic and diastolic blood pressure, resulting the heart to be in an overloaded hemodynamic state for a long time, and the body is often accompanied by neurohumoral response, which leads to myocardial cell hypertrophy, interstitial fibrosis, and LVH phenomenon [22]. The EH is a kind of vascular inflammation. The patient's left ventricular afterload increases, resulting in increased sST2 in cardiomyocytes and vascular endothelial cells. And increased sST2 inhibits the protective effect of Th2-type immune response on the myocardium, causing LVH. ST2 is the humoral marker in the genome group that is most susceptible to the mechanical tension of cardiomyocytes, and as a downstream product of ST2, sST2 has a significantly increased concentration in patients with acute or chronic heart failure and is closely related to LVH [23]. Because the increase of MMP-3 promotes the excessive degradation of collagen and the destruction of the collagen network structure, which makes the connection between the myocardial cells tend to loosen, the arrangement of myocardial cells is disordered, the wall of the myocardial ventricular thickens, the weight of the heart increases, and the normal interstitial structure disappears, leading to LVH. Some scholars have observed that, in the sheep model of compensatory left ventricular hypertrophy, a variety of MMPs including MMP-3 increased, collagen content decreased, and matrix remodeling increased [24]. In addition, the Gal-3 is an inflammatory signaling molecule, which plays an important role in the regulation of the body's inflammatory response in EH patients. The Gal-3 can regulate ventricular function, causing abnormal proliferation of myocardial cells, myocardial fibrosis, and decreased myocardial compliance, thereby impairing left ventricular function and causing LVH. Studies have found that, in animal experiments, the level of Gal-3 in rats has been significantly increased during the phase of compensatory myocardial hypertrophy. Gal-3 can induce the proliferation and differentiation of myocardial fibroblasts, promote the increase in the production of type I collagen, and lead to myocardial fibrosis and diastolic dysfunction [25].

## 5. Conclusion

The levels of sST2, MMP-3, and Gal-3 in the serum of EH patients increase with the aggravation of EH disease, and all are closely related to LVH. Dynamic detection of serum sST2, MMP-3, and Gal-3 levels can predict and judge ventricular remodeling in patients with EH to a certain extent, provide a new idea for early detection and prevention of LVH in patients with EH, thereby helping to reduce the complications of patients with EH, and improve the prognosis of the patients with EH. There are still some improvements to be made in this study, and the results of this study need to be confirmed by multicenter, large-sample and prospective studies, and it needs to be analyzed in conjunction with endpoint events, so as to have more clinical value. We need to supplement and improve this study in future studies.

## Figures and Tables

**Figure 1:** Comparison of the levels of sST2, MMP-3, and Gal-3 in the serum of the EH group and the control group. Note: compared with the control group, ^*∗*^*p* < 0.05.

**Figure 2:** Comparison of the levels of sST2, MMP-3, and Gal-3 in the serum with different level EH patients. Note: compared with the level 1 EH group, ^*∗*^*p* < 0.05; compared with the level 2 EH group, ^#^*p* < 0.05.

**Figure 3:** Comparison of the levels of sST2, MMP-3, and Gal-3 in the serum between the LVH group and the NLVH group. Note: compared with the NLVH group, ^*∗*^*p* < 0.05.

**Table 1:** Risk factors for the occurrence of LVH in patients with EH.

Influencing factors	*B* value	*SE* value	*Walds* value	*p* value	*OR* value	95% CI
Age	0.490	0.316	2.405	0.107	1.632	0.878–3.032
BMI	0.284	0.192	2.188	0.168	1.328	0.911–1.935
Systolic pressure	0.595	0.230	6.692	0.030	1.813	1.155–2.846
Diastolic pressure	0.511	0.243	4.422	0.034	1.667	1.035–2.683
Fasting blood glucose	0.621	0.455	1.880	0.183	1.860	0.762–4.539
TC	1.097	0.864	1.612	0.192	2.995	0.550–16.288
TG	1.162	0.690	2.836	0.095	3.196	0.826–12.359
sST2	1.873	0.545	11.811	0.005	6.208	2.236–18.938
MMP-3	1.264	0.487	6.736	0.029	3.540	1.362–9.193
Gal-3	1.375	0.469	8.595	0.016	3.955	1.577–9.916

**Table 2:** Correlation between the levels of serum sST2, MMP-3, Gal-3, and LVMI.

Item	sST2 (ng/mL)		MMP-3 (ng/mL)		Gal-3 (ng/mL)	
	*r* value	*p* value	*r* value	*p* value	*r* value	*p* value
LVMI	0.638	*p* < 0.01	0.446	0.029	0.597	*p* < 0.01

## Data Availability

The data used and/or analyzed during the current study are available from the corresponding author upon request.

## References

[1] Vallée A., Safar M. E., Blacher J. (2019). Essential hypertension: definitions, hemodynamic, clinical and therapeutic review. *Presse Medicale*.

[2] Liu D., Yi L., Sheng M., Wang G., Zou Y. (2020). The efficacy of tai chi and qigong exercises on blood pressure and blood levels of nitric oxide and endothelin-1 in patients with essential hypertension: a systematic review and meta-analysis of randomized controlled trials. *Evidence-based Complementary and Alternative Medicine*.

[3] Mahajan S., Feng F., Hu S. (2020). Assessment of prevalence, awareness, and characteristics of isolated systolic hypertension among younger and middle-aged adults in China. *JAMA Network Open*.

[4] Yildiz M., Oktay A. A., Stewart M. H., Milani R. V., Ventura H. O., Lavie C. J. (2020). Left ventricular hypertrophy and hypertension. *Progress in Cardiovascular Diseases*.

[5] Lovic D., Narayan P., Pittaras A., Faselis C., Doumas M., Kokkinos P. (2017). Left ventricular hypertrophy in athletes and hypertensive patients. *Journal of Clinical Hypertension*.

[6] Aimo A., Januzzi J. L., Bayes-Genis A. (2019). Clinical and prognostic significance of sST2 in heart failure. *Journal of the American College of Cardiology*.

[7] Zhang Z., Shen B., Cao X. (2017). Increased soluble suppression of tumorigenicity 2 level predicts all-cause and cardiovascular mortality in maintenance hemodialysis patients: a prospective cohort study. *Blood Purification*.

[8] Guizani I., Zidi W., Zayani Y. (2019). Matrix metalloproteinase-3 predicts clinical cardiovascular outcomes in patients with coronary artery disease: a 5 years cohort study. *Molecular Biology Reports*.

[9] Hu W., Wei R., Wang L., Lu J., Liu H., Zhang W. (2018). Correlations of MMP-1, MMP-3, and MMP-12 with the degree of atherosclerosis, plaque stability and cardiovascular and cerebrovascular events. *Experimental and Therapeutic Medicine*.

[10] Iacoviello M., Di Serio F., Rizzo C. (2019). Association between high Gal-3 serum levels and worsening of renal function in chronic heart failure outpatients. *Biomarkers in Medicine*.

[11] Martínez-Martínez E., Brugnolaro C., Ibarrola J. (2019). CT-1 (Cardiotrophin-1)-Gal-3 (Galectin-3) Axis in cardiac fibrosis and inflammation. *Hypertension*.

[12] Jones N. R., McCormack T., Constanti M., McManus R. J. (2020). Diagnosis and management of hypertension in adults: NICE guideline update 2019. *British Journal of General Practice*.

[13] Petrie J. R., Guzik T. J., Touyz R. M. (2018). Diabetes, hypertension, and cardiovascular disease: clinical insights and vascular mechanisms. *Canadian Journal of Cardiology*.

[14] Shenasa M., Shenasa H. (2017). Hypertension, left ventricular hypertrophy, and sudden cardiac death. *International Journal of Cardiology*.

[15] Kercheva M., Ryabova T., Gusakova A., Suslova T. E., Ryabov V., Karpov R. S. (2019). Serum soluble ST2 and adverse left ventricular remodeling in patients with ST-segment elevation myocardial infarction. *Clinical Medicine Insights: Cardiology*.

[16] Lotierzo M., Dupuy A. M., Kalmanovich E., Roubille F., Cristol J. P. (2020). sST2 as a value-added biomarker in heart failure. *Clinica Chimica Acta*.

[17] Parikh R. H., Seliger S. L., Christenson R., Gottdiener J. S., Psaty B. M., DeFilippi C. R. (2016). Soluble ST2 for prediction of heart failure and cardiovascular death in an elderly, community-dwelling population. *Journal of the American Heart Association*.

[18] Linssen P. B. C., Brunner-La Rocca H. P., Schalkwijk C. G. (2020). Serum matrix metalloproteinases and left atrial remodeling-the hoorn study. *International Journal of Molecular Sciences*.

[19] González G. E., Rhaleb N.-E., D’Ambrosio M. A. (2016). Cardiac-deleterious role of galectin-3 in chronic angiotensin II-induced hypertension. *American Journal of Physiology-Heart and Circulatory Physiology*.

[20] Sun Z., Zhang L., Li L. (2021). Galectin-3 mediates cardiac remodeling caused by impaired glucose and lipid metabolism through inhibiting two pathways of activating Akt. *American Journal of Physiology - Heart and Circulatory Physiology*.

[21] Stanton T., Dunn F. G. (2017). Hypertension, left ventricular hypertrophy, and myocardial ischemia. *Medical Clinics of North America*.

[22] Al-Sharifi A., Mingher H. M. (2019). Microalbuminuria and left ventricular hypertrophy in patients with essential hypertension. *Journal of the Pakistan Medical Association*.

[23] Kim M., Lee D. I., Lee J.-H. (2021). Lack of prognostic significance for major adverse cardiac events of soluble suppression of tumorigenicity 2 levels in patients with ST-segment elevation myocardial infarction. *Cardiology Journal*.

[24] Euler G., Locquet F., Kociszewska J. (2021). Matrix metalloproteinases repress hypertrophic growth in cardiac myocytes. *Cardiovascular Drugs and Therapy*.

[25] Wu Z. S., Lo J. J., Wu S. H. (2018). Early hyperbaric oxygen treatment attenuates burn-induced neuroinflammation by inhibiting the galectin-3-dependent toll-like receptor-4 pathway in a rat model. *International Journal of Molecular Sciences*.

